The article "Influence of the Driving Pressure on Mortality in ARDS Patients with or without Abdominal Obesity: A Retrospective Cohort Study" was published in 2022. Journal: Contrast Media Mol Imaging.

# Influence of the Driving Pressure on Mortality in ARDS Patients with or without Abdominal Obesity: A Retrospective Cohort Study

**DOI:** 10.1155/2022/1219666

**Published:** 2022-07-15

**Authors:** Shanshan Li, Bin Chen, Chaoyang Tong

**Affiliations:** Zhongshan Hospital, Fudan University, Shanghai 200032, China

## Abstract

**Objective:**

This study sets out to explore if the relationship between the driving pressure and hospital mortality in ARDS patients is influenced by body mass index (BMI) level or the presence of abdominal obesity.

**Methods:**

Data were extracted from an online database named “Multiparameter Intelligent Monitoring in Intensive Care III.” A total of 1556 patients were included and divided into four subgroups based on both BMI level (BMI ≥30 kg/m^2^ or BMI ＜30 kg/m^2^) and abdominal assessment. Driving pressure [i.e., the difference between plateau pressure and positive end-expiratory pressure (PEEP)] within 24 h of invasive mechanical ventilation was compared between survivors and nonsurvivors during hospitalization in each group. A logistic regression model was used for hospital mortality.

**Results:**

There were 1556 patients with mild-to-severe ARDS, 666 (42.80%) nonobese patients with nonabdominal obesity, 259 (16.65%) nonobese patients with abdominal obesity, 97 (6.23%) obese patients with nonabdominal obesity, and 534 (34.32%) obese patients with abdominal obesity. Driving pressure in nonobese patients with nonabdominal obesity was significantly lower in survivors (12.77 ± 4.53 cm H_2_O) than in nonsurvivors (14.26 ± 5.52 cm H_2_O, *p* < 0.01). On the contrary, in the other three groups, driving pressure was not significantly different between survivors and nonsurvivors. After a logistic multivariable regression analysis, in nonobese (BMI<30 kg/m^2^) patients with nonabdominal obesity, the driving pressure was independently associated with increased hospital mortality (OR: 1.04, 95% CI 1.00–1.09, *p* < 0.05) but not in the other three subgroups.

**Conclusion:**

Driving pressure is associated with increase in hospital mortality only in nonobese (BMI <30 kg/m^2^) patients with nonabdominal obesity.

## 1. Introduction

Obesity, a chronic disease that is increasing in prevalence globally, is a major contributor to poor health in most countries [1]. The acute respiratory distress syndrome (ARDS) is an acute and diffuse inflammatory condition of the lungs, characterized by hypoxaemia and bilateral pulmonary infiltrates. Different from nonobese patients, obese patients have a higher incidence of ARDS but may have a lower mortality risk [2, 3].

Mechanical ventilation is the main support for most of ARDS patients, which can also worsen lung injury [4–6]. Thus, the goal of ARDS therapy today is to improve oxygenation and prevent the occurrence of ventilator induced lung injury (VILI). The driving pressure [i.e., the difference between plateau pressure and positive end-expiratory pressure (PEEP)] determined by the quotient of the tidal volume and the respiratory system compliance was associated with higher mortality in ARDS [7], even in patients receiving extracorporeal membrane oxygenation [8]. However, conclusions from these studies cannot be extrapolated to all subgroups of patients with ARDS, especially those with elevated chest wall elastance, such as obese patients, and the obesity status could be a confounding factor in the relationship between driving pressure and mortality in overall ARDS patients. To our knowledge, there are very few clinical research works in regard to driving pressure in obese ARDS patients. Only Jong et al. reported the relationship between driving pressure during the first day of ventilation and 90-day mortality in obese patients with ARDS in 2018 [9]; however, their work did not take abdominal obesity into account.

Compliance of the chest wall in obesity is likely to be influenced by fat distribution. A larger change in chest wall compliance is observed when mass loading the upper abdomen and thorax than when mass loading the upper thorax [10]. Thus, it is of vital importance to reevaluate the association between mortality and obesity status considering the presence of abdominal fat in the invasive mechanical ventilation of ARDS patients. Our hypotheses were that mortality was correlated with driving pressure only in nonobese ARDS patients classified by BMI without abdominal obesity characterized by relatively high abdominal fat distribution, independent of BMI.

## 2. Methods

### 2.1. Study Design and Data Source

We conducted a retrospective cohort study, based on a freely available clinical database called the Multiparameter Intelligent Monitoring in Intensive Care III (MIMIC-III). It comprised deidentified health-related data associated with over 40,000 patients who stayed in critical care units of the Beth Israel Deaconess Medical Center between 2001 and 2012 [11]. The database is accessible to researchers who have completed a “protecting human subjects” training. The institutional review boards of the Massachusetts Institute of Technology (Cambridge, MA) and Beth Israel Deaconess Medical Center (Boston, MA) approved the establishment of the database. Thus, the consent was obtained for the original data collection but not specifically for this study. Data presented in this study were extracted by the author Li, who completed the online training course of the National Institutes of Health (certification number: 43513082). Data extraction was performed using PostgreSQL tools.

### 2.2. Study Population and Grouping Method

All the ARDS patients who were 18 years old or older without pregnancy and receiving invasive ventilation for at least 24 consecutive hours were included in the present investigation. Patients receiving ventilation through a tracheostomy cannula at any time during the first 24 h of ventilation and patients who were extubated or died during the first 24 h were excluded. For patients with multiple ICU and hospital admissions, we only included data from the first ICU admission and first hospital stay.

ARDS was identified based on the Berlin criteria [4]: (1) timing: onset within 1 week of a known clinical insult or new or worsening respiratory symptoms; (2) chest imaging: bilateral opacities, not fully explained by effusions, lobar/lung collapse, or nodules; (3) origin of edema: respiratory failure not fully explained by cardiac failure or fluid overload; and (4) oxygenation: oxygenation index (PaO_2_/FiO_2_ ratio) ≤300 mmHg with PEEP or continuous positive airway pressure (CPAP) ≥5 cmH_2_O.

Patients were assigned to one of the four subgroups. Grouping criteria were based on both body mass index (BMI) level, that is, BMI ≥30 kg/m^2^ for obese and BMI<30 kg/m^2^ for nonobese patients, in accordance with international standards [12], and abdominal assessment, that is, nonabdominal obesity and abdominal obesity, considering there were no data about waist circumference in MIMIC-III database.

### 2.3. Outcome Variables

The following information was extracted: (1) basic information: age, gender, BMI, race, comorbidity, type of admission, hospital or ICU length of stay (LOS), hospital mortality, sequential organ failure assessment score, simplified Acute Physiology Score II (SAPS II), systemic inflammatory response syndrome (SIRS) score, vasopressor use (including adenosine, norepinephrine, dopamine, dobutamine, and vasopressin), neuromuscular blocking agent (NMBA), and continuous renal replacement therapy (CRRT); (2) mechanical ventilation information: tidal volume, tidal volume/PBW (predicted body weight), peak pressure, plateau pressure, positive end-expiratory pressure (PEEP), driving pressure, and biologic parameters on day 1 [arterial PH, arterial partial pressure of oxygen (PaO_2_), oxygenation index (PaO_2_/FiO_2_ ratio), and arterial partial pressure of carbon dioxide (PaCO_2_)].

The primary endpoint was hospital mortality, defined as death during hospitalization. Secondary endpoints included ICU mortality, 28 d mortality, ICU length of stay (LOS), hospital LOS, and duration of invasive mechanical ventilation.

### 2.4. Statistical Analysis

Continuous variables are presented as the mean with SD or medians with their interquartile ranges and categorical variables as total number and percentage. Continuous variables were compared using Student's *t*-test or Wilcoxon's rank-sum test, and categorical variables were compared using *χ*^2^ or Fisher's exact test as appropriate. A logistic multivariable regression, selected as the analysis technique for all outcomes to account for factors that may influence outcomes, was conducted in different patient group, respectively. A stepwise backward elimination method with a significance level of 0.05 was used to build the final models. Potential multicollinearity was tested using a variance inflation factor, with a value ≥10 indicating multicollinearity. Goodness of fit was assessed for all logistic regression models. All analyses were performed using STATA MP 14.0 (USA). All tests were two sided, and a significance level of 0.05 was used.

### 2.5. Patient and Public Involvement

Patients were not involved in conduction of this research or its conception and design. We plan to disseminate the findings to the public and patients through the popular media and through the participating general practices.

## 3. Results

### 3.1. Population and Baseline Characteristics

The MIMIC-III database contained 58,976 ICU admissions of 46,520 unique patients. We excluded 34820 because the patients did not use invasive mechanical ventilation more than 24 h, 1222 for age below than 18 years (1222) or pregnancy (0), and 9462 because of insufficient data or having outliers. Only 1556 patients were included in this analysis, 384 nonsurvivors and 1172 survivors, establishing an initial mortality rate of 24.68%. The mean age was 63.28 ± 16.05 years, and 914 patients were male (58.74%).

Demographic characteristics of the survivors and nonsurvivors in overall patients or in each of four different subgroups determined by the BMI and abdominal assessment are presented in Table 1. Age, BMI, ARDS severity, SAPS II, SOFA, SIRS, vasopressor, NMBA, and CRRT showed significant differences among the survivors and nonsurvivors in overall patients (one-way ANOVA, all *p* < 0.01), while no significant differences in comorbidities were noted.

Ventilatory characteristics of the survivors and nonsurvivors are shown in Table 2. Driving pressure was significantly lower for survivors (13.56 ± 4.64) than for nonsurvivors (14.38 ± 5.30) (*p*=0.0066). When performing subgroup analyses, statistical differences among the survivors and nonsurvivors were only found in nonobese patients without abdominal obesity subgroup (12.77 ± 4.53 versus 14.26 ± 5.52, *p*=0.0012). In addition, the driving pressure difference between nonobese patients without abdominal obesity and obese patients with abdominal obesity subgroup was significant (13.18 ± 4.86 versus 14.47 ± 4.64, *p* < 0.0001) (Figure 1).

Crude outcomes are given in Table 3 for the four subgroups. The hospital mortality, ICU mortality, and 28 d mortality rate were not significantly different between patients with and without abdominal obesity. However, ICU LOS, hospital LOS, and duration of invasive mechanical ventilation were significantly shorter in the patients without abdominal obesity irrespective of BMI after adjusting for covariates.

To further explore the effect of driving pressure on the hospital mortality of ARDS patients, all the included patients were divided into four subgroups, and, after logistic multivariable regression analysis, the independent relationship between driving pressure and hospital mortality was demonstrated [OR = 1.04 (95% CI 1.00–1.09), *p*=0.027] (Table 4) in nonobese patients without abdominal obesity. However, no independent correlations were found in the other three subgroups [OR = 1.01 (95% CI 0.94–1.07), *p*=0.875 in Model 2; OR = 1.01 (95% CI 0.85–1.21), *p*=0.877 in Model 3; OR = 0.99 (95% CI 0.94–1.04), *p*=0.769 in Model 4].

## 4. Discussion

To the best of our knowledge, this is the first research to assess the association between driving pressure and mortality in ARDS specific patients who have an abdominal obesity with BMI greater or less than 30. The principal finding here was that driving pressure was independently related to mortality only in nonobese patients, classified by BMI level without abdominal obesity.

Very recently, a computational investigation performed by Saffaran et al. identified different strategies that minimized driving pressure or mechanical power consistently across pediatric and adult datasets and found that targeting driving pressure for minimization resulted in ventilator settings that also reduced mechanical power and modified mechanical power but not vice versa. Therefore, appropriate mechanical ventilation to decrease driving pressure is safer for mechanically ventilated patients than mechanical power [13]. Amato et al. using multilevel mediation analysis as a statistical tool found that driving pressure was most strongly associated with survival even in patients receiving “protective” plateau pressures and tidal volume [7]. A multicenter prospective cohort study published in JAMA confirmed these results and found that the increasing of driving pressure on the first day of ARDS was more relevant to hospital death than plateau pressure, and patients with a driving pressure greater than 14 cm H_2_O on day 1 of ARDS criteria had higher mortality rate [14]. Our results are largely consistent with those of previous studies. In this study, we did find statistically significant differences between survivors and nonsurvivors using one-way ANOVA, and the value of driving pressure was below 14 cm H_2_O for survivors. However, multivariate logistic regression analysis showed that driving pressure was not an independent prognostic factor for hospital death in overall ARDS patients. There are several possible causes for the discrepancy of the results between our previous study and this study. First, the sample size is relatively small. Second, it may be due to significant collinearity between independent variables in multivariate logistic regression analysis for overall ARDS patients. Our data identified driving pressure (odds ratio: 1.02; *p*=0.142); thus we further subgrouped the patients to decrease variance inflating factor (VIF) of independent variables. However, a retrospective observational analysis conducted by Schmidt showed that driving pressure was not associated with hospital death in non-ARDS mechanically ventilated patients [15].

In specific ARDS patients such as obese patients with ARDS, driving pressure is still not one size that can fit all. Obesity significantly interferes with respiratory system by direct mechanical changes as well as systemic inflammation [16]. Thus, the value of driving pressure found in the nonobese ARDS patients cannot be extrapolated to obese ARDS patients. Chiumello et al. evaluated the effect of the BMI in a group of ARDS patients on chest wall elastance, lung recruitability, and transpulmonary pressure. Meanwhile, obese ARDS patients did not show higher chest wall elastance compared with normal-weight patients [17]. Regretfully, there were very few research studies concerning the relationship between obese patients and driving pressure specifically. As far as we know, only recently Jong et al. published a study assessing the relationship between driving pressure during the first day of ventilation and 90-day mortality in obese patients classified by BMI with ARDS; the result demonstrated that driving pressure was not associated with 90-day mortality in obese ARDS patients [9], but two critical limitations should be noted. First, the obesity criteria were determined only based on BMI without considering the distribution of fat or the presence of abdominal fat. Second, this research did not distinguish the invasive mechanical ventilation of ARDS patients from noninvasive patients, probably owing to the relative small sample size. The value of driving pressure of nonobese patients (i.e., BMI <30 kg/m^2^) found in our research is in line with previous studies. But, in obese patients, in particular severely obese patients (i.e., BMI ≥40), the driving pressure was more than 14 cm H_2_O no matter in survivors or in nonsurvivors without statistically significant differences. Moreover, the driving pressure increased as BMI category increased. Furthermore, when patients were divided into four subgroups based on BMI level and abdominal assessment, statistically significant differences occurred between survivors and nonsurvivors only in nonobese patients with nonabdominal obesity subgroup, and driving pressure was independently associated with hospital mortality in this subgroup. A North Indian adolescent study reported that abdominal obesity was more prevalent than generalized obesity and showed increasing trend with age. Interestingly, over one-third of centrally obese adolescents were not obese by BMI criteria [18]. The main explanations of the differences observed between ARDS patients with and without abdominal obesity even in nonobese patients may be the following: For the vast majority of research works related to mechanical ventilation in obese ARDS patients, the obesity criteria were determined based on BMI only, which cannot reflect the body fat mass distribution or the presence of abdominal obesity, since the pattern of body fat distribution significantly influences the function of the respiratory system, likely via the direct mechanical effect of fat accumulation in the chest and abdominal regions; that is, the possible increase in chest wall elastance may modify the effects of the driving pressure on lung stress.

A relationship between higher BMI and longer lengths of stay but not ARDS mortality was reported by Gong et al. [19]. Similar to these results, Anzueto et al. [2] found that the obese patients were more likely to have significant complications during the course of ventilatory support including ARDS and acute renal failure, but there were no associations with increased duration of mechanical ventilation, length of stay, or mortality. The present findings differ from those reported in previous studies due to the different subgrouping method.

The results of this study suggest that driving pressure may not be appropriate to evaluate the severity of obese ARDS patients or nonobese patients with abdominal obesity; thus, we should focus not only on obesity but also on the distribution of fat. Predicted value equations for lung function testing have largely been developed from nonobese subjects, while a weight term is included in some lung function prediction equations; the association between body mass and lung function is influenced by obesity prevalence in the population [20, 21]. With no studies on the relationship between central obesity and driving pressure of mechanical ventilation, our results support the use of titrating PEEP by electrical impedance tomography or other indicators rather than driving pressure to monitor the obese ARDS patients or nonobese ARDS patients with abdominal obesity.

Some limitations exist in this study. First, the design was monocentric with a retrospective analysis, although this report was based on a large clinical database, MIMIC-III. Second, the abdominal obesity was based on abdominal assessment not abdominal circumference, due to missing abdominal girth data for ARDS patents in MIMIC-III. Third, although weight was determined on ICU admission, we cannot completely exclude the influence of fluid balance prior to ICU admission on the BMI.

## 5. Conclusion

Driving pressure is associated with increased hospital mortality only in nonobese (BMI <30 kg/m^2^) patients with nonabdominal obesity. We suspected that predefined ventilator settings that are similar for ARDS patients with and without abdominal obesity no matter BMI level may not be appropriate, since central obesity represents the massive load of the obese abdomen and the distribution of adipose tissue in the thoracic region reduce lung volume, impair the stability of the airways, and accelerate small airways collapse, thus inducing intrinsic positive end-expiratory pressure (PEEP). Thus, titrating PEEP to decrease driving pressure may be more reasonable for these patients.

## Figures and Tables

**Figure 1:** Values of driving pressure according to different grouping methods. Driving pressure was calculated as the difference between plateau pressure and PEEP on day 1 of mechanical ventilation. Group 1: nonobese patients without obesity; group 2: nonobese patients with obesity; group 3: obese patients without obesity; group 4: obese patients with obesity; values were given as mean. (1) Driving pressure was significantly lower in nonobese patients without abdominal obesity than in obese patients with abdominal obesity (13.18 ± 4.86 versus 14.47 ± 4.64, *p* < 0.0001). (2) In nonobese patients without abdominal obesity subgroup, driving pressure was significantly lower in survivors than in nonsurvivors (12.77 ± 4.53 versus 14.26 ± 5.52, *p*=0.0012). (3) In nonobese patients (i.e., with BMI ≥30 kg/m^2^), driving pressure was significantly lower in survivors than in nonsurvivors (13.06 ± 4.76 versus 14.25 ± 5.38, *p*=0.0024).

**Table 1:** Demographics of nonobese and obese patients with or without abdominal obesity.

Variable	Overall (*n* = 1556)		*p*	Nonobese patients without abdominal obesity (*n* = 666)		*p*	Nonobese patients with abdominal obesity (*n* = 259)		*p*	Obese patients without abdominal obesity (*n* = 97)		*p*	Obese patients with abdominal obesity (*n* = 534)		*p* value
	Survivors (*n* = 1172)	Nonsurvivors (*n* = 384)		Survivors (*n* = 482)	Nonsurvivors (*n* = 184)		Survivors (*n* = 198)	Nonsurvivors (*n* = 61)		Survivors (*n* = 78)	Nonsurvivors (*n* = 19)		Survivors (*n* = 414)	Nonsurvivors (*n* = 120)	
Age (years)	62.03 ± 15.98	67.09 ± 15.68	<0.0001	61.96 ± 17.12	67.48 ± 16.22	0.0002	66.62 ± 14.67	69.40 ± 16.41	0.2098	59.54 ± 18.40	67.89 ± 12.38	0.0641	60.38 ± 14.23	65.21 ± 14.88	0.0013
Male (*n* (%))	689 (58.79%)	225 (58.59)	0.946	297 (61.62%)	121 (65.76%)	0.323	110 (55.56%)	33 (54.10%)	0.841	49 (62.82%)	13 (68.42%)	0.2078	233 (56.28%)	58 (48.33%)	0.124
BMI (kg/m^2^)	29.93 ± 8.40	28.72 ± 7.46	0.0076	23.74 ± 3.41	23.62 ± 3.65	0.7086	26.51 ± 2.60	26.63 ± 2.54	0.7421	32.61 ± 2.51	33.90 ± 3.53	0.0676	38.27 ± 7.80	36.77 ± 6.43	0.033
Type of admission															
Elective (*n* (%))	103 (8.79%)	15 (3.91%)	0.003	41 (8.51%)	10 (5.43%)	0.149	15 (7.58%)	0 (0.00%)	0.044	2 (2.56%)	2 (10.53%)	0.203	45 (10.87%)	3 (2.50%)	0.005
Emergency (*n* (%))	1054 (89.93%)	366 (95.31%)		435 (90.25%)	174 (94.57%)		179 (90.40%)	60 (98.36%)		74 (94.87%)	17 (89.47%)		366 (88.41%)	115 (95.83%)	
Urgent (*n* (%))	15 (1.28%)	3 (0.78%)		6 (1.24%)	0 (0.00%)		4 (2.02%)	1 (1.64%)		2 (2.56%)	0 (0.00%)		3 (0.72%)	2 (1.67%)	
ARDS severity															
Mild	505 (43.09%)	130 (33.85%)	<0.001	214 (44.40%)	55 (22.89%)	0.001	81 (40.91%)	22 (36.07%)	0.492	38 (48.72%)	4 (21.05%)	0.072	172 (41.55%)	49 (40.83%)	0.339
Moderate	540 (46.08%)	186 (48.44%)		212 (43.98%)	92 (50.00%)		90 (45.45%)	27 (44.26%)		30 (38.46%)	11 (57.89%)		208 (50.24%)	56 (46.67%)	
Severe	127 (10.84%)	68 (17.71%)		56 (11.62%)	37 (20.11%)		27 (13.64%)	12 (19.67%)		10 (12.82%)	4 (21.05%)		34 (8.21%)	4 (12.50%)	
Other comorbidities															
HTN (*n* (%))	454 (38.74%)	145 (37.76%)	0.733	169 (35.06%)	66 (35.87%)	0.845	76 (38.38%)	22 (36.07%)	0.744	28 (35.90%)	8 (42.11%)	0.615	181 (43.72%)	49 (40.83%)	0.574
COPD (*n* (%))	130 (11.09%)	32 (8.33%)	0.124	50 (10.37%)	17 (9.24%)	0.663	24 (12.12%)	5 (8.20%)	0.395	7 (8.97%)	0 (0.00%)	0.339	49 (11.84%)	10 (8.33%)	0.281
CAD (*n* (%))	214 (18.26%)	69 (17.97%)	0.898	77 (15.98%)	30 (16.30%)	0.918	41 (20.71%)	20 (32.79%)	0.052	10 (12.82%)	2 (10.53%)	1.000	86 (20.77%)	17 (14.71%)	0.106
DM (*n* (%))	240 (20.65%)	83 (21.61%)	0.686	56 (11.62%)	27 (14.67%)	0.286	40 (20.20%)	9 (14.75%)	0.342	14 (17.95%)	7 (36.84%)	0.073	132 (31.88%)	40 (33.33%)	0.765
CKD (*n* (%))	152 (12.97%)	65 (16.93%)	0.052	52 (10.79%)	28 (15.22%)	0.116	31 (15.66%)	11 (18.03%)	0.052	6 (7.69%)	5 (26.32%)	0.022	63 (15.22%)	21 (17.50%)	0.545
Admission SAPS II	40.05 ± 14.00	50.44 ± 15.28	<0.0001	39.80 ± 13.46	50.47 ± 15.18	<0.0001	43.05 ± 14.13	52.02 ± 13.63	<0.0001	38.73 ± 12.42	57.95 ± 17.79	0.0002	39.54 ± 13.70	47.89 ± 15.08	<0.0001
Admission SOFA	5.88 ± 3.52	7.91 ± 4.25	<0.0001	5.61 ± 3.43	7.65 ± 4.27	<0.0001	6.50 ± 3.53	7.48 ± 4.14	0.0713	5.77 ± 3.34	11.16 ± 4.87	0.0001	6.00 ± 3.37	7.92 ± 3.88	<0.0001
Admission SIRS	3 (2–4)	3 (3–4)	<0.0001	3 (3–4)	3 (3–4)	0.0023	3 (2–4)	3 (3–4)	0.0582	3 (2–4)	4 (3–4)	0.0012	3 (2–4)	3 (3–4)	0.4403
Drug use															
Vasopressor	282 (24.06%)	214 (55.73%)	<0.001	103 (21.37%)	100 (54.35%)	<0.001	60 (30.30%)	35 (57.38%)	<0.001	13 (16.67%)	12 (63.16%)	<0.001	106 (25.60%)	67 (55.83%)	<0.001
NMBA	275 (23.46%)	123 (32.03%)	0.001	109 (22.61%)	56 (30.43%)	0.037	50 (25.25%)	22 (36.07%)	0.099	14 (17.95%)	3 (15.79%)	1.000	102 (24.64%)	42 (35.00%)	0.024
CRRT	59 (5.03%)	81 (21.09%)	<0.001	19 (3.94%)	22 (11.96%)	<0.001	14 (7.07%)	15 (24.59%)	<0.001	4 (5.13%)	11 (57.89%)	<0.001	22 (5.31%)	33 (27.50%)	<0.001

Values are given as mean ± SD, medians with their interquartile ranges, or number (%). BMI, body mass index; ARDS, acute respiratory distress syndrome; HTN, hypertension; COPD, chronic obstructive pulmonary disease; CAD, coronary arterial disease; DM, diabetes mellitus; CKD, chronic kidney disease; SAPS II, simplified acute physiology score II; SOFA, sequential organ failure assessment; SIRS, systemic inflammatory response syndrome; vasopressor, including adenosine, norepinephrine, dopamine, dobutamine, and vasopressin; NMBA, neuromuscular blocking agents; CRRT, continuous renal replacement therapy.

**Table 2:** Mechanical ventilation information on day 1 in nonobese and obese patients with or without abdominal obesity.

Variable	Overall (*n* = 1556)		*p*	Nonobese patients without abdominal obesity (*n* = 666)		*p*	Nonobese patients with abdominal obesity (*n* = 259)		*p*	Obese patients without abdominal obesity (*n* = 97)		*p*	Obese patients with abdominal obesity (*n* = 534)		*p* value
	Survivors (*n* = 1172)	Nonsurvivors (*n* = 384)		Survivors (*n* = 482)	Nonsurvivors (*n* = 184)		Survivors (*n* = 198)	Nonsurvivors (*n* = 61)		Survivors (*n* = 78)	Nonsurvivors (*n* = 19)		Survivors (*n* = 414)	Nonsurvivors (*n* = 120)	
Tidal volume (ml)	486.70 ± 104.50	481.00 ± 108.51	0.3582	473.65 ± 102.16	466.43 ± 115.20	0.4569	485.80 ± 95.82	475.08 ± 88.01	0.4373	497.12 ± 99.93	523.44 ± 154.13	0.4859	500.36 ± 110.26	499.62 ± 94.89	0.9419
Tidal volume/PBW (ml/kg)	7.57 ± 1.70	7.64 ± 1.89	0.5010	7.33 ± 1.65	7.22 ± 1.78	0.4398	7.57 ± 1.65	7.61 ± 1.57	0.8662	7.72 ± 1.53	8.77 ± 3.32	0.1935	7.82 ± 1.78	8.14 ± 1.74	0.0878
Number of patients (*n* (%)) ventilated with tidal volume															
≤8 ml/kg	654 (55.80%)	235 (61.20%)	<0.001	300 (62.24%)	127 (69.02%)	0.0010	109 (55.05%)	39 (63.93%)	0.0050	39 (50.00%)	11 (57.89%)	0.5040	206 (49.76%)	58 (48.33%)	0.0100
8.1–10 ml/kg	279 (23.81%)	94 (24.48%)		101 (20.95%)	31 (16.85%)		41 (20.71%)	19 (31.15%)		23 (29.49%)	3 (15.79%)		114 (27.54%)	41 (34.17%)	
10.1–12 ml/kg	58 (4.95%)	31 (8.07%)		12 (2.49%)	14 (7.61%)		14 (7.07%)	1 (1.64%)		4 (5.13%)	2 (10.53%)		28 (6.76%)	14 (11.67%)	
＞12 ml/kg	181 (15.44%)	24 (6.25%)		69 (14.32%)	12 (6.52%)		34 (17.17%)	2 (3.28%)		12 (15.38%)	3 (15.79%)		66 (15.94%)	7 (5.83%)	
Peak pressure (cmH_2_O)	21.35 ± 7.40	24.40 ± 8.25	<0.0001	20.57 ± 7.18	23.60 ± 8.16	<0.0001	20.77 ± 7.78	23.54 ± 7.55	0.0151	21.34 ± 6.84	26.53 ± 11.45	0.0717	22.53 ± 7.43	25.72 ± 8.03	0.0001
Plateau pressure (cmH_2_O)	20.36 ± 5.25	22.14 ± 6.06	<0.0001	19.06 ± 5.19	21.56 ± 5.83	<0.0001	20.50 ± 5.42	21.92 ± 5.96	0.0830	19.80 ± 4.64	24.05 ± 7.97	0.0365	21.92 ± 4.92	22.85 ± 6.06	0.1248
PEEP (cmH_2_O)	5 (5–10)	7.5 (5–10)	0.0001	5 (5–8)	5 (5–10)	0.0003	5 (5–10)	6 (5–10)	0.1785	5 (5–10)	8 (5–15)	0.0021	8 (5–10)	7.5 (5–11)	0.3984
Number of patients (*n* (%)) ventilated with PEEP															
≤5 cm H_2_O	682 (58.19%)	189 (49.22%)	0.002	315 (65.35%)	95 (51.63%)	0.005	118 (59.60%)	30 (49.18%)	0.4250	49 (62.82%)	5 (26.32%)	0.0010	200 (48.31%)	59 (49.17%)	0.1540
5.1–7.5 cm H_2_O	11 (0.94%)	3 (0.78%)		5 (1.04%)	1 (0.54%)		2 (1.01%)	1 (1.64%)		0 (0.00%)	0 (0.00%)		4 (0.97%)	1 (0.83%)	
7.6–10 cm H_2_O	334 (28.50%)	117 (30.47%)		119 (24.69%)	60 (32.61%)		53 (26.77%)	20 (32.79%)		24 (30.77%)	7 (36.84%)		138 (33.33%)	30 (25.00%)	
>10 cm H_2_O	145 (12.37%)	75 (19.53%)		43 (8.92%)	28 (15.22%)		25 (12.63%)	10 (16.39%)		5 (6.41%)	7 (36.84%)		72 (17.39%)	30 (25.00%)	
Driving pressure (cmH_2_O)	13.56 ± 4.64	14.38 ± 5.30	0.0066	12.77 ± 4.53	14.26 ± 5.52	0.0012	13.77 ± 5.21	14.21 ± 4.97	0.559	13.52 ± 4.01	13.75 ± 4.67	0.826	14.39 ± 4.45	14.76 ± 5.26	0.4784
Biologic parameters on day 1															
Arterial PH	7.39 ± 0.84	7.36 ± 0.11	<0.0001	7.39 ± 0.09	7.35 ± 0.11	<0.0001	7.39 ± 0.08	7.36 ± 0.13	0.0515	7.38 ± 0.09	7.31 ± 0.11	0.0046	7.38 ± 0.08	7.38 ± 0.10	0.6138
PaO_2_ (mmHg)	93.82 ± 31.43	90.52 ± 30.68	0.0724	93.39 ± 31.78	90.67 ± 35.65	0.3406	91.49 ± 29.39	89.89 ± 27.13	0.7046	97.82 ± 38.88	88.42 ± 29.25	0.3264	94.68 ± 30.41	90.93 ± 23.96	0.1581
PaCO_2_ (mmHg)	44.46 ± 13.09	42.66 ± 13.12	0.0199	43.60 ± 13.37	43.63 ± 14.21	0.98	42.44 ± 12.02	40.64 ± 10.66	0.2938	41.21 ± 8.20	47.42 ± 15.33	0.1025	47.04 ± 13.59	41.47 ± 11.90	0.0001
PaO_2_/FiO_2_ ratio	187.10 ± 63.24	170.15 ± 67.62	<0.0001	188.41 ± 64.43	164.36 ± 70.04	<0.0001	182.75 ± 63.58	170.22 ± 66.68	0.1847	185.67 ± 68.38	153.92 ± 74.90	0.078	187.91 ± 60.77	181.57 ± 62.10	0.3167

Values are given as mean ± SD, medians with their interquartile ranges, or number (%). PEEP, positive end-expiratory pressure; PBW, predicted body weight.

**Table 3:** Comparisons of outcomes between patients with and without abdominal obesity.

Variable	Nonobese patients without abdominal obesity (*n* = 666)	Nonobese patients with abdominal obesity (*n* = 259)	*p*	Obese patients without abdominal obesity (*n* = 97)	Obese patients with abdominal obesity (*n* = 534)	*p* value
Hospital mortality (*n* (%))	184 (27.63%)	61 (23.55%)	0.207	19 (19.59%)	120 (22.47%)	0.528
ICU mortality (*n* (%))	156 (23.42%)	52 (20.08%)	0.274	19 (19.59%)	95 (17.79%)	0.672
28 d mortality (*n* (%))	179 (26.88%)	55 (21.24%)	0.076	16 (16.49%)	109 (20.41%)	0.373
Hospital LOS (days)	12.63 (7.5–20.75)	13.96 (9.04–24.88)	0.0027	11.54 (7.63–16.5)	13.71 (8.29–22.58)	0.0431
ICU LOS (days)	6.19 (3.13–11.92)	8.79 (4.13–14.5)	0.0002	4.92 (2.75–8.04)	7.94 (4.04–14.58)	<0.0001
Duration of invasive mechanical ventilation (days)	4.21 (2.38–8.63)	5.96 (3–11.04)	0.0001	3.96 (2.13–6.08)	5.48 (2.83–9.92)	0.0002

Values are given as medians with their interquartile ranges or number (%). LOS, length of stay.

**Table 4:** Adjusted ORs of driving pressure for hospital mortality by logistic multivariable regression analysis in four subgroups.

Variable	OR	95% CI	*p* value	VIF
Model 1: correlation between driving pressure and hospital mortality in nonobese patients without abdominal obesity				
Driving pressure	1.04	1.00–1.09	0.027	5.13
ARDS severity	1.52	1.16–2.00	0.003	
Vasopressor	2.93	1.98–4.34	<0.001	
SAPS II	1.04	1.03–1.06	<0.001	

Model 2: correlation between driving pressure and hospital mortality in nonobese patients with abdominal obesity				
Driving pressure	1.01	0.94–1.07	0.875	4.79
Vasopressor	2.04	1.05–3.96	0.036	
SAPS II	1.05	1.02–1.08	0.001	
SOFA	0.88	0.78–0.98	0.025	

Model 3: correlation between driving pressure and hospital mortality in obese patients without abdominal obesity				
Driving pressure	1.01	0.85–1.21	0.877	4.98
SOFA	1.279	1.04–1.57	0.018	
SIRS	2.69	1.02–7.11	0.046	
Age	1.06	1.01–1.12	0.018	
CRRT	15.26	2.06–112.9	0.008	

Model 4: correlation between driving pressure and hospital mortality in obese patients with abdominal obesity				
Driving pressure	0.99	0.94–1.04	0.769	2.91
Vasopressor	2.19	1.34–3.57	0.002	
SOFA	1.07	1.00–1.15	0.044	
Age	1.03	1.01–1.04	0.001	
CRRT	4.27	2.24–8.14	<0.001	

ARDS, acute respiratory distress syndrome; SAPS II, simplified acute physiology score II; SOFA, sequential organ failure assessment; SIRS, systemic inflammatory response syndrome; vasopressor, including adenosine, norepinephrine, dopamine, dobutamine, and vasopressin; NMBA, neuromuscular blocking agents; CRRT, continuous renal replacement therapy.

## Data Availability

The full dataset is available from the corresponding upon request. However, reanalysis of the full data needs to be approved by MIMIC-III Institute.

## References

[1] Collaboration N. C. D. R. F. (2016). Trends in adult body-mass index in 200 countries from 1975 to 2014: a pooled analysis of 1698 population-based measurement studies with 19.2 million participants. *Lancet*.

[2] Anzueto A., Vivar F. F., Esteban A. (2011). Influence of body mass index on outcome of the mechanically ventilated patients. *Thorax*.

[3] O’Brien J. M., Philips G. S., Ali N. A., Aberegg S. K., Marsh C. B., Lemeshow S. (2012). The association between body mass index, processes of care, and outcomes from mechanical ventilation: a prospective cohort study. *Critical Care Medicine*.

[4] Force A. D. T., Ranieri V. M., Rubenfeld G. D. (2012). Acute respiratory distress syndrome: the Berlin definition. *JAMA*.

[5] Fan E., Del Sorbo L., Hodgson E. C. (2017). An official American thoracic society/European society of intensive care medicine/society of critical care medicine clinical practice guideline: mechanical ventilation in adult patients with acute respiratory distress syndrome. *American Journal of Respiratory and Critical Care Medicine*.

[6] Slutsky A. S., Ranieri V. M. (2013). Ventilator-induced lung injury. *New England Journal of Medicine*.

[7] Amato M. B., Meade M. O., Brochard A. S. (2015). Driving pressure and survival in the acute respiratory distress syndrome. *New England Journal of Medicine*.

[8] Neto A. S., Schmidt M., Azevedo L. C. P. (2016). Associations between ventilator settings during extracorporeal membrane oxygenation for refractory hypoxemia and outcome in patients with acute respiratory distress syndrome: a pooled individual patient data analysis. *Intensive Care Medicine*.

[9] Jong A. D., Cossic J., Monet C. (2018). Impact of the driving pressure on mortality in obese and non-obese ARDS patients: a retrospective study of 362 cases. *Intensive Care Medicine*.

[10] Sharp JT., Henry JP., Sweany SK., Meadows W R., Pietras R J. (1964). Effects of mass loading the respiratory system in man. *Journal of Applied Physiology*.

[11] Johnson A. E., Pollard T. J., Lehman L. w. H. (2016). MIMIC-III, a freely accessible critical care database. *Scientific Data*.

[12] (1998). Executive summary of the clinical guidelines on the identification, evaluation, and treatment of overweight and obesity in adults. *Archives of Internal Medicine*.

[13] Saffaran S., Das A., Laffey J. G., Hardman J. G., Yehya N., Bates D. G. (2020). Utility of driving pressure and mechanical power to guide protective ventilator settings in two cohorts of adult and pediatric patients with acute respiratory distress syndrome: a computational investigation. *Critical Care Medicine*.

[14] Bellani G., Laffey J. G., Fan T. (2016). Epidemiology, patterns of care, and mortality for patients with acute respiratory distress syndrome in intensive care units in 50 countries. *JAMA*.

[15] Schmidt M. F. S., Amaral A., Fan E., Rubenfeld G. D. (2018). Driving pressure and hospital mortality in patients without ARDS. *Chest*.

[16] Brazzale D. J., Pretto J. J., Schachter L. M. (2015). Optimizing respiratory function assessments to elucidate the impact of obesity on respiratory health. *Respirology*.

[17] Chiumello D., Colombo A., Mietto I. (2016). Effect of body mass index in acute respiratory distress syndrome. *British Journal of Anaesthesia*.

[18] Solanki D. K., Walia R., Gautam A., Misra A., Aggarwal A. K., Bhansali A. (2020). Prevalence of abdominal obesity in non-obese adolescents: a North Indian adolescent study. *Journal of Pediatric Endocrinology & Metabolism*.

[19] Gong M. N., Bajwa E. K., Thompson B. T., Christiani D. C. (2010). Body mass index is associated with the development of acute respiratory distress syndrome. *Thorax*.

[20] Roca J., Rodriguez Roisin R., Cobo E., Burgos F., Perez J., Clausen J. L. (1990). Single-breath carbon monoxide diffusing capacity prediction equations from a mediterranean population. *American Review of Respiratory Disease*.

[21] Bruschi C., Cerveri I., Zoia M. C. (1992). Reference values of maximal respiratory mouth pressures: a population-based study. *American Review of Respiratory Disease*.

